# Berberine Alleviates Gastroesophageal Reflux-Induced Airway Hyperresponsiveness in a Transient Receptor Potential A1-Dependent Manner

**DOI:** 10.1155/2022/7464147

**Published:** 2022-05-09

**Authors:** Bo Zou, Chaofan Cao, Yue Fu, Dianzhu Pan, Wei Wang, Lingfei Kong

**Affiliations:** ^1^Institute of Respiratory Diseases, The First Hospital of China Medical University, Shenyang City, Liaoning Province, China; ^2^Department of Respiratory and Critical Care Medicine, The Fourth Affiliated Hospital of China Medical University, Shenyang City, Liaoning Province, China; ^3^Department of Respiratory Medicine, The Second Affiliated Hospital of Shenyang Medical College, Shenyang City, Liaoning Province, China; ^4^Department of Respiratory Medicine, The First Affiliated Hospital of Jinzhou Medical University, Jinzhou City, Liaoning Province, China

## Abstract

**Background:**

To investigate the beneficial effect of berberine on gastroesophageal reflux-induced airway hyperresponsiveness (GERAHR) and explore the underlying mechanism.

**Methods:**

Coword cluster analysis and strategic coordinates were used to identify hotspots for GERAHR research, and an online tool (STRING, https://string-db.org/) was used to predict the potential relationships between proteins. Guinea pigs with chemically induced GERAHR received PBS or different berberine-based treatments to evaluate the therapeutic effect of berberine and characterize the underlying mechanism. Airway responsiveness was assessed using a plethysmography system, and protein expression was evaluated by western blotting, immunohistochemical staining, and quantitative PCR analysis.

**Results:**

Bioinformatics analyses revealed that TRP channels are hotspots of GERAHR research, and TRPA1 is related to the proinflammatory neuropeptide substance P (SP). Berberine, especially at the middle dose tested (MB, 150 mg/kg), significantly improved lung function, suppressed inflammatory cell infiltration, and protected inflammation-driven tissue damage in the lung, trachea, esophagus, and nerve tissues in GERAHR guinea pigs. MB reduced the expression of TRPA1, SP, and tumor necrosis factor-alpha (TNF-*α*) in evaluated organs and tissues. Meanwhile, the MB-mediated protective effects were attenuated by simultaneous TRPA1 activation.

**Conclusions:**

Mechanistically, berberine was found to suppress GERAHR-induced upregulation of TRPA1, SP, and TNF-*α* in many tissues. Our study has highlighted the potential therapeutic value of berberine for the treatment of GERAHR.

## 1. Introduction

Gastroesophageal reflux disease (GERD), a common global disease with increasing prevalence, has become a burden on public healthcare [1]. GERD causes various symptoms, and chronic cough is one of the most commonly observed symptoms. Airway hyperresponsiveness (AHR) has been postulated as one of the etiologies of chronic cough in GERD patients. However, current clinical outcomes for this disease and its complications are still not satisfactory. Thus, it is necessary to characterize the pathogenesis of this disorder and develop more effective therapeutic drugs.

The etiology of gastroesophageal reflux-induced airway hyperresponsiveness (GERAHR) is multifactorial, and one of the primary mechanisms involves esophageal-bronchial nerve reflex-mediated neurogenic inflammation [2]. Accumulating evidence has revealed the role of transient receptor potential (TRP) channel subfamily *A* member 1 (TRPA1), one of the TRP channel families, in GERAHR pathogenesis. TRPA1 antagonists have been shown to attenuate AHR and its symptoms, while the agonists were reported to escalate inflammation and exacerbate symptoms of AHR [3, 4]. In addition, upregulation of TRPA1 in the sensory nerve terminals has been observed in the respiratory tract upon exposure to stimuli such as endogenous and exogenous agonists [5, 6]. On the other hand, several peptides released from airway sensory nerve cells, including substance P (SP) and neurokinin A (NKA), have been shown to contribute to airway inflammation *via* promoting the release of proinflammatory cytokines [7, 8]. Moreover, recent studies have demonstrated that TRPA1 regulates the production of proinflammatory neuropeptides, including SP, calcitonin gene-related peptide (CGRP), and NKA [9]. Therefore, TRPA1 may be associated with the progression of GERAHR in an SP-dependent manner.

Berberine is a benzylisoquinoline alkaloid isolated from many medicinal plants [10]. Berberine exhibits an anti-inflammatory effect by inhibiting the production of tumor necrosis factor-alpha (TNF-*α*), interleukin-6 (IL-6), and monocyte chemoattractant protein 1 (MCP-1) [11]. More importantly, recent experimental evidence has revealed that berberine attenuated neurogenic inflammation in the gastrointestinal tract mainly by suppressing the production of SP [12]. Therefore, it is highly possible that berberine can also protect the respiratory tract during GERAHR from neurogenic inflammation through downregulating SP. In addition, berberine has been shown to inhibit the activity of TRPV1 [13], another member of the TRP superfamily. It has been well-documented that TRPV1 and TRPA1 are structurally and functionally related [14]. Therefore, it is possible that berberine can protect against neurogenic inflammation by suppressing TRPA1 and downregulating SP production in the respiratory tract during GERAHR.

Hence, the therapeutic effects of berberine were investigated in a guinea pig model of GERAHR. In addition, pulmonary function after treatment with berberine was evaluated to determine the therapeutic outcome. Furthermore, we investigated the underlying mechanism whereby berberine-mediated TRPA1 inhibition leads to a suppressed inflammatory response.

## 2. Materials and Methods

### 2.1. Research Hotspots in GERAHR Identified Using Coword Cluster Analysis and Strategic Coordinates

#### 2.1.1. Data Collection

A primary literature search (term: gastroesophageal reflux airway hyperresponsiveness (GERAHR)) was performed for all relevant studies published between 2007 and 2017. Two reviewers independently reviewed and selected articles based on the predetermined inclusion/exclusion criteria. Finally, 711 related research articles were selected, and data were collected and saved as previously described [15].

The Bibliographic Item Co-Occurrence Matrix Builder version 2.0 (BICOMB 2.0 software; 202.118.40.8/bc) was used to identify and sort keywords from the selected articles [16]. Keywords with a cumulative frequency of occurrence ≥38% were considered hotspots in GERAHR research.

The relationship among high-frequency keywords was determined by performing two or more statistical calculations based on the number of times those words appeared in the same paper. BICOMB was used to generate a 62 × 62 text matrix, where the content of the rows was article sources and the content of the columns was high-frequency keywords. gCLUTO software (version 1.0; glaros.dtc.umn.edu/gkhome/cluto/gcluto/download) with adjusted settings was then used to perform bicluster analysis [15] using the BICOMB-generated matrix. The clustering method was repeated bisectionally, and the clustering criterion function was I2 [15]. Different numbers of clusters were used to repeat the analysis to obtain ideal external and internal similarities to determine the optimal number of clusters. The high-frequency and high-frequency bifocal results of the MeSH articles were visualized by Alpine and Matrix. Using the semantic relationship between MeSH terminology and the content of representative papers in each group, the basic framework and processing of GERAHR research hotspots were extracted and analyzed. In this way, GERAHR hotspots were obtained.

#### 2.1.2. Coword Strategic Coordinates

Strategic coordinates were used to describe interrelationships and interfield interactions in GERAHR-related research. Density (the vertical axis) represents the category's ability to maintain and develop itself [17]. Centrality (the horizontal axis) reflects the degree of interactions between the keywords from each category [18]. The greater the number and intensity of associations between one subject and other categories, the more central the subject to the entire area of research. Based on the high-frequency keyword cooccurrence matrix and the results of coword cluster analysis, the centrality and density of each category were calculated. The basic framework of GERAHR research for all categories was then mapped, and current international developmental trends in the field of GERAHR studies were analyzed using strategic coordinates.

### 2.2. Bioinformatic Prediction of TRPA1-SP Interaction

The potential interaction between TRPA1 and SP was predicted using online tools (STRING, https://string-db.org/) following methods provided in a previous study [19].

### 2.3. Establishment of GERAHR

#### 2.3.1. Establishment of the Guinea Pig Model of GERAHR

GERAHR was induced by repeated esophageal infusion of hydrochloric acid (HCl) in guinea pigs [20]. Fifty-six healthy male albino guinea pigs weighing 300–400 g (6–8 weeks old) were obtained from the Beijing Weitong Lihua Experimental Animal Technological Company. Eight guinea pigs were randomly assigned to the control group, while the rest of the animals received HCl for the induction of GERAHR. First, guinea pigs were anesthetized with an intraperitoneal injection of ketamine (50 mg/kg). Then, animals were placed supine, and a 5 F catheter was inserted into the middle and lower esophagus through the mouth (intubation depth: 11–13 cm). Each animal was perfused (flow rate: 26 mL/h) with HCl (0.1 mol/L containing 0.5% pepsin) or sterile distilled water for 20 min once a day for a total of 14 days. Experiments were carried out according to the National Institute of Health Guide for Care and Use of Laboratory Animals and were approved by the Bioethics Committee of China Medical University.

#### 2.3.2. Treatment

GERAHR guinea pigs were randomly assigned to one of six groups based on the treatment received [21]: PBS group (PBS-treated GERAHR guinea pig), LB group (low-dose berberine-treated GERAHR guinea pig, 75 mg/kg), MB group (medium-dose berberine-treated GERAHR guinea pig, 150 mg/kg), HB group (high-dose berberine-treated GERAHR guinea pig, 300 mg/kg), MB + agonists allyl isothiocyanate group (AITC, w203408, Sigma-Aldrich; medium-dose berberine + AITC-treated GERAHR guinea pig), and HC-030031 group (Selleck, S2918, 2 mg/kg; HC-030031-treated GERAHR guinea pig). Guinea pigs that received water during GERAHR establishment were used as control animals (normal). Berberine (Solarbio Technology, Beijing, China) dissolved in PBS was administered to each GERAHR guinea pig via oral gavage using an animal feeding bulbous-ended needle (20 ga). Guinea pigs from each group received the treatments as indicated for three consecutive days, and the animals were then subjected to further studies.

### 2.4. Measurement of Airway Responsiveness

Twenty-four hours following the last treatment, the breathing curve of guinea pigs from each group were depicted using a whole-body plethysmography system (Emka Company, France) [22]. Then, pulmonary function parameter (pulmonary enhanced pause, Penh, reflects airway resistance) was measured after inhalation of gradually increasing concentrations of aerosolized methacholine (Mch; baseline, 0, 3.12, 6.25, 12.5, 25, 50, and 100 *μ*g/kg) as previously described [22].

### 2.5. Collection and Detection of BALF

Bronchoalveolar lavage (BAL) was performed as described previously [23]. In brief, immediately after measuring pulmonary function, BAL was performed by instillation of sterile PBS (3 mL) into the lung through the trachea. The total number of cells in the bronchoalveolar lavage fluid (BALF) was counted using a hemacytometer. Next, the BALF was centrifuged (7 min, 2,000 rpm), and cells were resuspended and left to adhere to a slide overnight. The adhered cells were subjected to hematoxylin and eosin (H & E) staining. The percentages of monocytes, eosinophils, and neutrophils in the BALF were determined by counting 400 leukocytes in randomly selected areas of the slide using a light microscope.

### 2.6. Histological Analysis

Three days following treatment, animals were euthanized, and tissues were harvested and fixed in 4% paraformaldehyde for subsequent paraffin embedding and sectioning prior to H & E staining to observe pathological changes as previously described [24]. Meanwhile, immunohistochemistry (IHC) was performed to detect the expression of TRPA1 (1 : 200, Novus, USA), SP (1 : 100 Abcam, Cambridge, UK), and TNF-*α* (1 : 100 Santa Cruz, USA) according to a previous study [25]. The staining intensity was estimated with Image-Pro Plus software (Media Cybernetics) by experienced technicians blinded to the study [25].

### 2.7. Western Blotting Analysis

The collected tissues were homogenized and lysed in radioimmunoprecipitation assay (RIPA) buffer supplemented with proteinase inhibitors (B14001, Bimake) for 30 min at 4°C followed by centrifugation (12,000 rpm, 30 min, 4°C). Solubilized proteins were separated in a 10% gel by sodium dodecyl sulfate-polyacrylamide gel electrophoresis (SDS-PAGE) and transferred to polyvinylidene fluoride (PVDF) membranes (Millipore, MA, USA). Next, membranes were incubated with primary antibodies at 4°C overnight against TRPA1 (1 : 400, Abcam) and glyceraldehyde 3-phosphate dehydrogenase (GAPDH; 1 : 1,000, Abcam) as the internal control. The next day, membranes were washed and incubated with secondary antibodies (1 : 5,000, ZSGB-BIO) at room temperature for 1 hour. Membranes were then developed with ClarityTM and Clarity MaxTM Western ECL Substrates (BIO-RAD) and visualized in the MicroChemi 4.2 (DNR Bio-Imaging Systems) imaging system. Protein bands were quantified using ImageJ software.

### 2.8. Quantitative Reverse Transcription-Polymerase Chain Reaction (qRT-PCR)

Total RNA from tissue was extracted using RNAiso Plus (Code No. 9108, TAKARA) and reverse transcribed into complementary DNA (cDNA) with a cDNA synthesis kit (RR047A, TAKARA Bio Inc.). Subsequently, TB Green™ Premix Ex Taq™ II (RR820A, Clontech Laboratories, Inc., A TaKaRa Bio Company) was used to quantify the mRNA expression levels on the Opticon® System (Bio-Rad, Hercules, CA). Primers for genes of interest were designed and synthesized by TaKaRa, and the sequences were as follows: TRPA1-F 5′-CAGCGGTTCTTCTTGTGAAGTG-3′, TRPA1-R 5′-GTTTGGGTTTGGATGCTTTGTTG-3′; GAPDH-F 5′-GAGAAA-CCGGCCAAATACGA-3′, GAPDH-R 5′-GTAAGAAGGTGAAAACTGCGAC-3′; SP-F 5′-GACCAGATCAAGGAGGCGCT-3′, SP-R 5′-TACCCGTTTTGCCCTACGACT-3′. GAPDH served as the internal reference, and the fold changes were calculated using the 2-ΔΔCt method.

### 2.9. Statistical Analysis

Statistical analyses were performed using a two-tailed Student's *t*-test for unpaired observations or a one-way analysis of variance (ANOVA) using SPSS software (version 23.0, IBM). The data were presented as mean ± standard error of the mean (SEM) of at least three independent experiments. *p* values < 0.05 were considered statistically significant.

## 3. Results

### 3.1. Bicluster Analysis of High-Frequency Words and Strategic Coordinates of GERAHR Categories

The BICOMB and bicluster analysis results identified 62 high-frequency keywords as hotspots in GERAHR research, as reflected by the visualization matrix (Figure 1(a)) and mountain map (Figure 1(b)). In addition, the 62 hotspots were categorized into four clusters (categories 1–4):

- Category 1: Studies on the mechanism of GERAHR
- Category 2: Models of GERAHR
- Category 3: Research on the pharmacological regulation of TRP channels
- Category 4: Clinical research on GERAHR

The density and centrality of each category are shown in Figure 1(c), and the basic framework for each study category is shown in Figure 1(d). As displayed in Figure 1(d), categories 3 and 4 have low density suggesting that our knowledge in these categories needs to be improved, which compelled us to study the connection between GERAHR and TRP family members.

### 3.2. STRING Analysis

Although accumulating evidence has linked TRPA1 expression and the production of the proinflammatory neuropeptide, SP, in various diseases and organs, the underlying molecular activities have not been defined [9]. In the current study, the STRING analysis filled this knowledge gap by revealing potential regulatory relationship between TRPA1 and SP. The data showed that TRPA1 was associated with tachykinin 1 (Tac1), which encodes SP [26]. Moreover, the result also unveiled signaling routes by which TRPA1 could regulate SP production. Together, these findings suggested how TRPA1 regulates SP expression and proposed the possibility that berberine may exert an effect on the TRPA1/SP axis to modulate the progression of GERAHR.

### 3.3. Results of Animal Experiments

#### 3.3.1. Berberine Promotes the Recovery of Mch-Induced Airway Hyperresponsiveness *In Vivo*

The guinea pig model of GERAHR was established to assess the therapeutic efficacy of berberine. Then, control and treated GERAHR guinea pigs underwent Mch challenge, and the lung function parameter termed Penh was measured to determine the airway resistance.  Figure 2(a) highlights no significant differences in Penh values in the animals of each group at baseline. However, the Penh values in the MB group were significantly lower than the PBS group with 25 *μ*g/kg of Mch. After stimulation with 25 *μ*g/kg Mch in the PBS group, the guinea pigs experienced severe dyspnea and could not receive a higher dose of Mch, whereas the control and MB-treated guinea pigs were able to tolerate higher doses of Mch.

To measure whether berberine can affect airway responsiveness, guinea pigs were challenged with sequentially increased concentrations of Mch. The breath of the animals was recorded using a noninvasive pneumatometer. The result revealed that, at basal condition, GERAHR guinea pigs exhibited extended expiration phages compared with normal ones. On the other hand, we noticed that, when there was no Mch, MB could restore GERAHR-related expiration elongation, while this effect could be compromised by TRPA1 agonist (AITC), while in the presence of Mch challenge, Mch resulted in a prolonged expiration phase in guinea pigs. Meanwhile, Mch-mediated extended expiration was more obvious in GERAHR animals compared with control guinea pigs. However, MB significantly attenuated Mch-mediated breathing difficulties in GERAHR animals compared with PBS. Moreover, this protective effect could be reversed by TRPA1 activation (Figure 2(a), left panel). Furthermore, the guinea pigs' airway responsiveness was noted, as reflected by the Penh value, and was elevated along with increasing Mch concentrations. Importantly, our data suggested that MB significantly reduced the Mch-elevated airway responsiveness in guinea pigs. Additionally, the MB-restored airway responsiveness could be abolished by simultaneous TRPA1 activation (Figure 2(a)).

#### 3.3.2. Berberine Inhibits Tissue Inflammation and Improves Tissue Structure

Studies have shown that GERAHR can cause inflammation in the esophagus and airway [27]. Thus, we next explored the total and differential cell counts in the BALF. The results revealed that the immune cell count in the BALF from guinea pigs in all GERAHR groups was increased compared with that in the normal control group. Moreover, compared with LB and HB treatments, MB significantly attenuated the accumulation of inflammatory cells (Figure 2(b)). Furthermore, these data suggested that MB was very effective in inhibiting the infiltration of all immune cells studied, including neutrophils, eosinophils, and monocytes, when compared to LB and HB treatments (Figures 2(c)–2(e)). These findings suggest that berberine, especially at the middle dose, possesses the therapeutic potential for treating GERAHR by suppressing the inflammatory response.

Next, the histological changes in tissues affected by GERAHR were investigated. In the control group, no tissue damage was observed in the lung, trachea, esophagus, and spinal cord tissue. However, infiltration of inflammatory cells was observed in all tissues from guinea pigs experiencing GERAHR (Figures 3(a)–3(d)). In the PBS group, inflammatory cell infiltration and alveolar wall thickening were observed in the lung (Figure 3(a)). However, administering berberine mitigated the accumulation of inflammatory cells and reduced the alveolar wall thickening. Importantly, MB achieved the best outcome. In the trachea, GERAHR guinea pigs from the PBS group exhibited loss of epithelium, accumulation of inflammatory cells at the denuded area, and vascular congestion and dilation (Figure 3(b)). Interestingly, these HCl-induced adverse effects were alleviated by berberine treatment, especially MB. The pathohistological changes were then evaluated in the esophagus. Epithelial hyperkeratosis, papillae hypertrophy, basal cell hyperproliferation, and squamous cell expansion were noted (Figure 3(c)). The above changes were lessened in the berberine groups, and importantly, the MB group had the most noticeable improvement. Furthermore, the inflammatory cell infiltration in the spinal cord was the most severe in the PBS group, while the MB group had the least immune cell infiltration (Figure 3(d)). More importantly, we found that GERAHR guinea pigs treated with a selective TRPA1 inhibitor, HC-030031, exhibited therapeutic outcomes comparable to berberine in the evaluated organs.

Therefore, our findings demonstrated that berberine protected tissues from inflammation-related damage by suppressing the infiltration of immune cells. Moreover, MB displayed the highest therapeutic efficacy. Furthermore, our findings also indicated that MB achieved a similar therapeutic effect as TRPA1 inhibition.

#### 3.3.3. Berberine Alleviates Tissue Inflammation in a TRPA1-Dependent Manner

To investigate the mechanism by which MB alleviated GERAHR-associated tissue damage in guinea pigs, the expression of TRPA1 in the lung, C7-T5 dorsal root ganglia (C7-T5), trachea, and esophagus was evaluated. The results revealed that MB significantly repressed the expression of TRPA1 compared with the PBS group in all tissues (Figures 4(a) and 4(b)). Of note, TRPA1 can control the release of SP [9], which plays an important role in the initiation and progression of neurogenic inflammation [8]. Therefore, it is possible that berberine-mediated TRPA1 suppression ultimately leads to a reduction in SP, which would protect the tissues from inflammation and damage. The results of the qRT-PCR analysis showed that, compared with the PBS group, guinea pigs in the MB group had significantly inhibited expression of SP in the lung, C7-T5, trachea, and esophagus (Figure 4(c)).

In addition, IHC analysis was also conducted to evaluate lung expression of SP and TNF-*α*. It was observed that the levels of SP (Figure 4(d)) and TNF-*α* (Figure 4(e)) were lower in the MB group compared to the PBS group. Interestingly, TRPA1 inhibition (HC-030031) also reduced the production of SP and TNF-*α* in the lung (Figures 4(d) and 4(e)). In parallel, the expression of TRPA1 in C7-T5 tissue was assessed, and the same result was observed (Figure 4(f)). These data support the speculation that berberine suppresses tissue inflammation by suppressing TRPA1.

It has been well documented that HC-030031, the selective TRPA1 inhibitor, can completely block the cough caused by a TRPA1 stimulant (isothiocyanate) *in vivo* [28]. Therefore, to gain insight into the mechanisms of MB-suppressed neuroinflammation, a TRPA1 agonist (AITC) was combined with MB to treat GERAHR, followed by qRT-PCR, IHC, and H & E analyses of the tissues. As a result, treatment with MB resulted in a significant reduction of TRPA1, which could be abolished by AITC, in the lung (Figures 5(a) and 5(d)), C7-T5 (Figures 5(a) and 5(e)), trachea, and esophagus (Figure 5(a)) compared to the PBS group, as reflected by the results of the qRT-PCR and IHC analysis. Meanwhile, it was also discovered that MB significantly reduced the production of TNF-*α* and SP in the lung of GERAHR guinea pigs compared to PBS, and this MB-mediated suppression could be neutralized by AITC (Figures 5(b) and 5(c)). Furthermore, H & E staining of the lungs also indicated that the therapeutic effect of MB was attenuated by AITC (Figure 5(f)).

In conclusion, these data revealed that the anti-inflammatory effects of berberine at least partially depend on its inhibitory role in the expression of TRPA1, which regulates the expression of proinflammatory factors in damaged tissues.

## 4. Discussion

GERAHR is one of the common causes of chronic cough [2]. So far, proton pump inhibitors are the standard therapy for GERAHR. However, approximately 30% of patients do not respond to this treatment [29]. Thus, it is necessary to thoroughly understand the pathogenesis and develop novel drugs for this disease. In this study, our bioinformatic analysis and *in vivo* study identified widely studied but underdeveloped areas in GERAHR research and revealed the therapeutic effects and an underlying mechanistic effect of berberine for the treatment of GERAHR.

Currently, bibliometric analyses are increasingly used to evaluate and review the status and trends in a particular field. For instance, this approach has been utilized to explore cancer research trends and evaluate potential drug targets [30, 31]. However, to the best of our knowledge, no bibliometric study focusing on GERAHR research has been reported. In the current study, the bibliometric analysis enabled us to test our hypothesis in the most well-demonstrated GERAHR model *in vivo* [20], which has added a layer of repeatability to our study. More importantly, our analysis showed that studies in category 3 focus on the regulation of TRP channels, and those in category 4 aim to explore clinical research relating to GERAHR, such as its treatment. However, our findings also indicate that our knowledge of these aspects is still limited. Therefore, results from the bibliometric analysis directed our attention in this study to the therapeutic approach for GERAHR and its potential regulatory effects on TRP family members, particularly TRPA1.

Although increasing evidence has emphasized the connection between TRPA1 and SP in disease pathogenesis, the underlying molecular mechanisms are still unclear. In this study, online database examination revealed that TRPA1 is associated with Tac1, which encodes SP [26]. Moreover, the data mining also predicted the potential signaling pathway by which SP expression could be regulated by TRPA1. In addition, TRPA1 and SP have long been associated with various disorders, including skin inflammation, neuropathic pain, and colitis [9]; however, their connection to GERAHR has not been elucidated. Therefore, we speculated that the TRPA1/SP axis might contribute to the pathogenesis of GERAHR. Of note, this study also revealed a gap between bench and bedside studies, indicating that more attention should be devoted to this area of research. The results suggest that the current therapeutic approaches, including medication and surgery, are insufficient to achieve a satisfactory outcome [29, 32]. Based on these analyses, we examined the therapeutic effects of berberine on GERAHR *in vivo*.

It has been reported that inhibiting TRPA1 suppresses airway inflammation and hyperresponsiveness in mice [28]. Meanwhile, it was speculated that berberine could suppress TRPA1 to mitigate the inflammatory response and resolve airway hyperresponsiveness. Therefore, to test if TRPA1 is an effector of berberine, gain-of-function assays were performed by activating TRPA1 in the current study. We have found that, compared to treatment with PBS, berberine significantly restored lung function upon stimulation with Mch, which was consistent with a previous study [33]. However, this effect was neutralized by a TRPA1 agonist (AITC). Consistent with this study, AITC has been shown to elicit airway inflammation and hyperresponsiveness [34]. These findings suggest that berberine exerts its function through the regulation of TRPA1. As TRPA1-mediated neurogenic inflammation is considered the primary mechanism of GERAHR [2], the inflammatory status of the airway was investigated by evaluating the infiltrated immune cells in the BALF. In guinea pigs with GERAHR, we observed significantly elevated inflammatory cell infiltration, as reflected by increased neutrophils, eosinophils, and monocytes in the BALF. Interestingly, berberine (all doses) significantly reduced the activation and infiltration of neutrophils, the critical mediator of airway inflammation. More importantly, MB significantly reduced the infiltration of all detected immune cell types in the BALF, including neutrophils, eosinophils, and monocytes. In alignment with our findings, the effects of berberine on inflammatory cell infiltration have also been observed in liver and airway inflammation [33, 35].

Also investigated were the histological changes in GERAHR-affected tissues. It was found that TRPA1 was upregulated in the lung, trachea, C7-T5, and esophagus in GERAHR animals. Along with the elevated TRPA1, SP and TNF-*α* were also increased, which likely contributed to tissue damage. These findings indicate a TRPA1/SP/TNF-*α* axis in GERAHR pathogenesis, which aligns with a previous study [36]. Meanwhile, compared to PBS, it was observed that berberine alleviated tissue damage and reduced inflammatory cell infiltration in the lung, trachea, and esophagus. In parallel, berberine also reduced the expression of TRPA1, SP, and TNF-*α* in these organs. However, the protective effects of berberine on tissue damage, immune cell infiltration, and proinflammatory mediator secretion could be reduced by AITC, a TRPA1 agonist. More importantly, the TRPA1 inhibitor HC-030031 also caused a comparable therapeutic effect in GERAHR guinea pigs. Importantly, HC-030031 is highly selective and does not affect other TRP family members such as the TRPVs or TRPCs [28]. Therefore, these data suggested that inhibiting TRPA1 could alleviate GERAHR-associated damage, while activating TRPA1 could exaggerate GERAHR-associated damage, which sheds light on the role of TRPA1 in GERAHR pathogenesis. Furthermore, these data indicated that berberine could attenuate inflammation and inflammation-associated damage of GERAHR *in vivo*. Consistent with these findings, the anti-inflammatory effects of berberine have been reported in previous studies [35, 37]. Together, these data revealed that berberine protected guinea pigs from GERAHR in a TRPA1-dependent manner.

It has been documented that berberine also exerts an inhibitory effect on other TRP family members such as TRPV1, TRPV3, and TRPC5 [13, 38]. Furthermore, TRPV1 has been shown to colocalize with TRPA1 in sensory neurons and is functionally related to TRPA1 in lung inflammation [39]. Therefore, it is reasonable to speculate that berberine can exert protective effects on TRPV1-associated pathways. However, it has been shown that relief of airway inflammation and airway hyperresponsiveness could be successfully achieved using a specific TRPA1 inhibitor (HC-030031) [40]. The data from the current study have also shown that HC-030031 successfully protected guinea pigs from GERAHR-mediated tissue damage and reduced the production of proinflammatory mediators, which was comparable to the effects of berberine. In addition, TRPA1 and TRPV1 have been shown to be coexpressed in various cell types, including sensory nerves [14], and the functional interaction between these two molecules has been previously described [14]. Therefore, it is difficult to dissect the independent functional roles of TRPA1 and TRPV1. An increasing amount of research has been conducted to investigate the cross-talk between TRPA1 and TRPV1, but the results are far from conclusive. For instance, TRPA1 has been demonstrated to sensitize TRPV1 [41], and conversely, TRPV1 has been reported to sensitize TRPA1 [42]. Moreover, it has also been documented that activating TRPA1 is sufficient to trigger the release of SP in nerves [43]. Therefore, it is suggested that, although TRPA1 and TRPV1 are colocalized and are able to cross-talk, they can perform their functions independently from one another.

However, we still cannot deny that certain therapeutic effects observed in this study could be caused by berberine-mediated TRPV1 inhibition. As such, this is one of the limitations of the current study. Investigation into whether and how TRPV1 is involved in the scenario of GERAHR treatment is being actively pursued as a component of our future research. There are other limitations to the current study. Firstly, whether berberine also affects other TRP family members that mediate the immune responses needs to be further explored. Secondly, how berberine regulates TRPA1 expression was not thoroughly dissected. For instance, our bioinformatic analysis revealed that TRPA1 is associated with SP through MAPK14, but the underlying molecular activities were not thoroughly investigated. Lastly, whether berberine also regulates the release of SP and TNF-*α* in a TRPA1-independent manner needs further investigation.

## 5. Conclusions

In conclusion, we provided a macroscopic overview of GERAHR that will help researchers grasp current trends and improve their understanding of the development of fundamental topics within the field. Our experiments showed that berberine alleviates GERAHR in a TRPA1-dependent manner.

## Figures and Tables

**Figure 1:** Results of bioinformatic analyses reflecting research hotspots and protein-protein interactions of TRPA1 in GERAHR. (a) The visualization matrix created from a cluster analysis of high-frequency subject words related to GERAHR using gGLUTO software. Color depth reflects the importance of the keywords within the literature. (b) The mountain map created from a cluster analysis of high-frequency keywords related to GERAHR. (c) Density and centrality of multiple keywords in GERAHR. (d) Strategic coordinates of various coword categories in GERAHR. Numbers 1, 2, 3, and 4 in this figure represent categories 1, 2, 3, and 4, respectively. (e) The interaction between TRPA1 and SP predicted by STRING.

**Figure 2:** Effect of berberine on airway responsiveness and differential cell counts in BALF following exposure to Mch. (a) Mch breathing curve at different concentrations in guinea pigs. (b–e) Analysis of the total cell counts (b) and percentages of neutrophils (c), eosinophils (d), and monocytes (e) in BALF (*n* = 8; ^*∗*^*p* < 0.05 versus PBS).

**Figure 3:** Effects of berberine on the tissue morphology in lung, trachea, esophagus, and spinal cord. H & E staining was performed to evaluate tissue morphology, tissue damage, and infiltration of inflammatory cells in the lung (a), trachea (b), esophagus (c), and spinal cord (d) of guinea pigs under the indicated treatments (*n* = 8; scale bars, 30 *μ*m).

**Figure 4:** Effects of berberine on TRPA1 expression and lung inflammation. (a) and (b) Representative images and quantitative results of western blot analysis evaluating the expression of TRPA1 in the lung, C7-T5, trachea, and esophagus exposed to indicated treatments. (c) Results of qRT-PCR determining mRNA level of SP in different tissues under indicated conditions. (d)–(e) Representative images of IHC analysis exploring the expression of SP (d) and TNF-*α* (e) in lung tissue of guinea pigs under indicated conditions. (f) Representative images of IHC analysis showing TRPA1 expression in the C7-T5 tissue. (*n* = 3; ^*∗*^*p* < 0.05 versus PBS; ^*∗∗*^*p* < 0.01 versus PBS).

**Figure 5:** AITC restored berberine-mediated inhibition of TRPA1 expression. (a) qRT-PCR analysis determined the expression of TRPA1 in the lung, C7-T5, trachea, and esophagus tissues of guinea pigs from indicated groups. (b–e) Representative IHC images and quantitative results showing lung expression of TNF-*α* (b), SP (c), and TRPA1 (d), and the expression of TRPA1 (e) in C7-T5 in guinea pigs from indicated groups. (f) Representative images of H & E staining evaluating the lung tissue structure of guinea pigs from indicated groups (*n* = 8; ^*∗*^*p* < 0.05 versus PBS; scale bars, 30 *μ*m).

## Data Availability

The datasets generated and analyzed during the present study are available from the corresponding author upon reasonable request.

## Abbreviations

GERD: Gastroesophageal reflux disease
GERAHR: Gastroesophageal reflux-induced airway hyperresponsiveness
BALF: Bronchoalveolar lavage fluids
H & E: Hematoxylin and eosin
WB: Western blotting
IHC: Immunohistochemistry
qRT-PCR: Quantitative reverse transcription-polymerase chain reaction
TRP: Transient receptor potential
AHR: Airway hyperresponsiveness
SP: Substance P
Tac1: Tachykinin 1
NKA: Neurokinin A
TRP: Transient receptor potential
TRPA1: Transient receptor potential channel subfamily A member 1
CGRP: Calcitonin gene-related peptide
TNF-*α*: Tumor necrosis factor-alpha
IL-6: Interleukin-6
MCP-1: Monocyte chemoattractant protein 1
BICOMB 2.0: The Bibliographic Item Co-Occurrence Matrix Builder version 2.0
AITC: Allyl isothiocyanate
BAL: Bronchoalveolar lavage
SDS-PAGE: Sodium dodecyl sulfate-polyacrylamide gel electrophoresis
PVDF: Polyvinylidene fluoride
cDNA: Complementary DNA
DRG: Dorsal root ganglion
MB: Medium-dose berberine
LB: Low-dose berberine
HB: High-dose berberine
Mch: Methacholine
PBS: Phosphate-buffered saline
C-T: Cervical, thoracic
C7-T5: Dorsal root ganglia C7-T5
Penh: Pulmonary enhanced pause.
